This article has been retracted.

# Treatment of Trigeminal Neuralgia With Stereotactic Radiosurgery Improved Symptoms of Morbihan Syndrome

**DOI:** 10.7759/cureus.20774

**Published:** 2021-12-28

**Authors:** Laura Burgess, Layth Mula-Hussain, Shawn Malone

**Affiliations:** 1 Department of Radiology, Division of Radiation Oncology, University of Ottawa, Ottawa, CAN; 2 Department of Radiology, Division of Radiation Oncology, The Ottawa Hospital Research Institute, Ottawa, CAN; 3 Department of Radiation Oncology, Sultan Qaboos Cancer Centre, Muscat, OMN

**Keywords:** neuropathic pain treatment, stereotactic radiosurgery (cyberknife®), morbihan syndrome, trigeminal neuralgia, stereotactic radiosurgery srs

## Abstract

Trigeminal neuralgia (TN) is a neuropathic pain disorder characterized by paroxysmal pain in the maxillary and mandibular regions of the face. Morbihan syndrome is a disease that classically presents with dermatologic findings, including progressive facial edema and erythema. There are no previous reports of the onset of trigeminal neuralgia with Morbihan syndrome or previous reports describing improvement in symptoms of Morbihan syndrome with treatment of trigeminal neuralgia. We describe the case of a 62-year-old female who presented with trigeminal neuralgia and shortly thereafter developed significant facial edema and was diagnosed with Morbihan syndrome. The neuralgia was refractory to medical management and was effectively treated with stereotactic radiosurgery (SRS). This coincided with an improvement in her Morbihan syndrome that is now controlled following stereotactic radiosurgery and continued lymphatic massage.

## Introduction

Trigeminal neuralgia (TN) is a chronic neuropathic pain disorder that classically presents with paroxysms of shock-like or stabbing pain that is spontaneous and elicited by innocuous stimuli to a region of the face [1]. Specifically, triggered paroxysmal pain is reported in up to 99% of patients [2,3]. Most commonly, it is secondary to intracranial vascular compression of the trigeminal nerve root. Other causes include trauma and neurologic disease (e.g., multiple sclerosis or tumors) that compromise the nerve [1]. Additionally, in approximately 10% of cases, there is no apparent cause for the neuralgia.

Morbihan syndrome is a rare disease with dermatologic features including non-depressive edema and erythema of the upper two-thirds of the face [4]. The syndrome is progressive in nature and does not regress spontaneously. It was first described in 1957 by Robert Degos, who observed the features in a farmer in Morbihan, France [5]. Marked facial edema tends to spread slowly and regionally and commonly involves the glabella, eyelids, and cheeks [4]. Its evolution is initially fluctuating but becomes more permanent with time, leading to significant facial disfigurement.

Herein, we review a patient with severe TN who later developed Morbihan syndrome. Following stereotactic radiosurgery (SRS), the patient had improvement in both the TN and the clinical symptoms of Morbihan syndrome.

## Case presentation

A 62-year-old female presented with a three-year history of right-sided facial pain involving the maxillary and mandibular branches of the trigeminal nerve (CNV). The pain was characteristic of TN with extreme, sporadic sharp stabbing and burning pain in the CNV2 and CNV3 distributions. The patient was seen by neurology in consultation. Her pain was triggered by light touch and eating. The patient had a brief response to neuralgia medications; however, she became refractory to medical therapy within a year. Additionally, the patient developed significant side effects from medical therapy, including fatigue, memory loss, and cognitive dysfunction. She endorsed that the pain was debilitating in nature. She was unable to perform activities of daily living (ADLs) and she became socially withdrawn from friends and family.

Approximately one year after her diagnosis of TN, she developed intermittent right-sided facial edema that progressed to intermittent bilateral facial edema. The edema was nonpitting and involved her bilateral cheeks and eyes. She had associated skin erythema. The facial edema progressed and became more persistent. The patient was seen by dermatology in consultation and was diagnosed clinically with Morbihan syndrome. She was started on isotretinoin and prednisone without clinical improvement.

The patient was seen in consultation by radiation oncology for consideration of SRS for her TN. Her past medical history was remarkable for TN (three-year duration), fibromyalgia, migraine headaches, asthma, restless leg syndrome, and alopecia areata. She had no history of trauma or injury to the trigeminal nerve. In addition, there was no history of multiple sclerosis or degenerative diseases. At the time of assessment, she had failed medical management for the TN with trials of pregabalin, gabapentin, topiramate, and oxcarbazepine. Topiramate relieved her migraine headaches, but it had no effect on her TN. She suffered a generalized rash from oxicarbazepine. On examination, she had marked facial edema. She was neurologically intact with a normal cranial nerve examination, normal motor power in her extremities, and normal cerebellar testing. Brain MRI (T1 volumetric interpolated breath-hold examination [VIBE], T2, fluid-attenuated inversion recovery and constructive interference in steady-state sequences [CISS]) did not reveal any abnormalities in the brain, skull base, or along the course of the trigeminal nerves. There was no evidence of vessel impingement on the trigeminal nerve, tumor in the skull base, or cerebellopontine angle.

In January 2021, the patient was treated with a single-fraction SRS to a dose of 60 Gy on CyberKnife (SRS plan shown in Figure 1). At the time of SRS, she was not on neuralgia medications due to intolerance of medical therapy. Several hours post-treatment, the patient developed a mild right-sided headache. She had no associated nausea, emesis, or ataxia. The headache was managed successfully with a short course of dexamethasone (4 mg by mouth daily for 10 days).

**Figure 1:** SRS plan on cyberKnife with (A) axial T1 VIBE post-gadolinium contrast; (B) axial CISS; (C) sagittal CISS images showing dose distribution. SRS: stereotactic radiosurgery, VIBE: volumetric interpolated breath-hold examination, CISS: constructive interference in steady-state sequence.

Two months after completion of SRS, her TN dramatically improved, with only rare episodes of mild neuralgia. In addition, her facial edema had significantly improved at this point. Other than the SRS, she had not received any active medical therapy for her Morbihan syndrome. Three months after SRS, she began treatment with gentle lymphatic massage for her residual facial edema. The massage therapy, along with her previous SRS, resulted in a marked improvement in her symptoms of Morbihan syndrome. She no longer has persistent edema and facial erythema. She has occasional episodes of mild edema in her bilateral cheeks which resolves with lymphatic massage.

At 11 months' follow-up after SRS, her TN pain remains significantly improved. She has no numbness or anesthesia dolorosa following SRS. She now performs all of her ADLs and has become interactive with friends and family. She experiences rare pain flares that can be controlled with simple analgesics. She also finds that the facial edema caused by Morbihan syndrome remains significantly improved. If the edema flares, it can now be effectively managed with gentle lymphatic massage.

## Discussion

Morbihan syndrome is a rare dermatologic condition characterized by profound facial edema. Patients typically present with significant swelling of the upper two-thirds of their faces. The edema can be so severe that it can result in disfigurement and visual field deficits [6]. Other common features include facial flushing, telangiectasia, papules, nodules, and granulomas [7]. The edema is thought to be secondary to poor lymphatic flow resulting from either chronic inflammation or lymphatic obstruction [8]. Histologically, this appears as the destruction of elastic connective tissue in perivascular tissue and the exudation of fluid [4,9].

Treatment effectiveness for Morbihan syndrome is inconsistent. Current treatment strategies tend to focus on the use of antibiotics (e.g., doxycycline), corticosteroids, and isotretinoin-based therapies. There is increased efficacy with a combination approach rather than single treatment modalities [8]. Other treatments include lymphatic massage, X-ray radiotherapy, antihistamines and interferon-gamma injections, but these often fail to resolve symptoms, or the symptoms may quickly recur [9,10].

Our patient presented with Morbihan syndrome approximately one year after the onset of symptoms of TN. Her symptoms were progressive in nature and resulted in significant cosmetic disfigurement. She had significant pain relief two months after stereotactic radiosurgery for her TN. Of interest, in this case, she also had marked improvement in her facial edema at the same time she noted relief from her neuralgia. She previously had no clinical benefit from a combination of corticosteroids and isotretinoin. The patient has noted benefit from gentle lymphatic massage.

Morbihan syndrome is so uncommon that it is only reported in case studies [6,11-13]. No previous case reports link the syndrome to TN or show improvement in symptoms following treatment of TN with SRS. There are reports of the use of superficial X-ray radiotherapy in the treatment of Morbihan syndrome, but with little effect [9,10].

Some recent studies have suggested the importance of inflammation in neuropathic pain [14-16]. However, the role of inflammation in TN remains unclear. Yao et al. recently investigated the level of inflammatory biomarkers in patients with TN versus normal controls [17]. The levels of white blood cells, neutrophils, monocytes, neutrophil/lymphocyte ratio, and monocyte/lymphocyte ratio were increased in TN patients compared to normal control subjects. Their research suggests that inflammation could have an important role in the progression and etiology of TN. We also know that agents such as isotretinoin, used in the treatment of Morbihan syndrome, are thought to be effective thanks to their immunomodulatory and anti-inflammatory properties [18,19]. We postulate that successful treatment of TN with SRS in our patient may have reduced the inflammatory process and helped to attenuate the symptoms of the Morbihan syndrome, but more research is needed to determine how SRS is able to stimulate such responses.

## Conclusions

In summary, there are no previously published case reports describing the onset of TN with Morbihan syndrome or describing improvement in symptoms of Morbihan syndrome with treatment of TN. We presented a case herein of a patient whose facial edema started one year after symptoms of TN. The neuralgia was refractory to medical management and was effectively treated with SRS. This coincided with an improvement in her Morbihan Syndrome that is now controlled following SRS and continued lymphatic massage.
